# Changes in power generation performance of an undershot cross-flow-type hydraulic turbine in an irrigation channel due to snow masses passing through the rotor

**DOI:** 10.1016/j.heliyon.2023.e20833

**Published:** 2023-10-13

**Authors:** Eiichi Satou, Tomomi Uchiyama, Kotaro Takamure, Toshihiko Ikeda, Tomoko Okayama, Tomoaki Miyazawa, Daisuke Tsunashima

**Affiliations:** a Faculty of Engineering, Niigata Institute of Technology, 1719 Fujihashi, Kashiwazaki, Niigata, 945-1195, Japan; b Institute of Materials and Systems for Sustainability, Nagoya University, Furo-cho, Chikusa-ku, Nagoya, 464-8601, Japan; c Faculty of Engineering, Shinshu University, 4-17-1 Wakasato, Nagano, 380-8553, Japan; d Faculty of Regional Development, Taisho University, 3-20-1 Nishi-Sugamo, Toshima-ku, Tokyo, 170-8470, Japan; e Chuetsu Kogyo Inc., 2-5-29 Matunami, Kashiwazai, Niigata, 945-0011, Japan

**Keywords:** Hydraulic turbine of undershot cross-flow type, Irrigation channel, Snow masses, Turbine performance

## Abstract

This study is focused on the development of a microhydraulic turbine that can stably and efficiently generate electricity even in channel where snow masses frequently flow down. A hydraulic turbine of an undershot cross-flow type was installed in an irrigation channel, and the change in the turbine performance was measured when spherical snowballs were released one by one from the upstream. The observation of the snowballs passing through the turbine was also conducted. Consequently, the variations in the power generated by the rotor were classified into three modes based on the motion of the snowballs, and could be organized by the ratio of the snowballs' cross-sectional area to the product of the rotor width and blade interval. Furthermore, the emergence of the power output overshoot phenomenon, in which the power output temporarily increases compared to clear water when the rotor restarts after stopping, was identified, and the relationship between the amount of loss when the rotor stops and that of electric energy gained during the overshoot was clarified. Certain guidelines for the installation of the undershot cross-flow type in irrigation channels of snowy regions was successfully obtained.

## Nomenclature

B: Rotor width m
Cp: Power output coefficient -
D: Rotor diameter m
d: Diameter of the snowball m
*E* ($E_{+}$, $E_{-}$): Electric energy J
Eˆ: Recovery rate of electric energy -
H: Depth of the irrigation channel m
H0: Water level at position $S_{1}$ when the turbine is not installed m
$H_{1}$ ($H_{10}$): Water level at position $S_{1}$ when the turbine is installed m
L: Blade spacing m
Ms: Mass flowrate of the snowball kg/s
Mw: Water mass flowrate kg/s
*m*: Number of snowballs per release -
*N* ($N_{0}$): Rotational speed rpm
n: Number of blades -
*P* ($P_{0}$): Power output of the generator W
R: Radius of the inside corner of the channel bottom mm
RL: Road resistor of the generator, Ω
*t* (Δ*t*, $t_{1}$, $t_{2}$, $t_{3}$, $t_{4}$): Time s
T0: Rotor rotational period at $N_{0}$ s
W: Width of the irrigation channel m
U0: Flow velocity in the irrigation channel when turbine is not installed m/s
V: Effective voltage V
β: Inlet angle of the blade °
λ: Tip speed ratio of the rotor -
ρw: Density of water kg/m^3^

## 1 Introduction

Hydropower is one of the oldest renewable energy sources in use today, and its application is expected to increase steadily in the future [1]. Recently, small-scale hydro-energy-based power generation from small rivers has garnered significant attention [2], [3]. This is because its power generation does not require large facilities, such as dams and water pipelines, and exerts a lower environmental impact. Furthermore, this small scale power generation can be a disaster-resistant distributed power source that enables local production for local consumption. Unused hydro-energy in irrigation channels, industrial drains, and water supply facilities is actively utilized to achieve carbon-neutral targets and the Sustainable Development Goals [4], [5], [6]. Small hydraulic turbines (hereinafter called “microhydraulic turbines”), such as cross-flow [7], [8], [9], [10], [11], [12], [13], [14], [15], [16], propeller [1], [17], [18], [19], [20], [21], [22], [23], [24], [25], [26], Savonius [27], [28], [29], [30], [31], Darrieus [32], [33], [34], and impulse types [35], [36], [37], have been developed for power generation, depending on the flow conditions. Regarding cross-flow turbines with high efficiency potential, the effects of the nozzle geometry [7], water-fall thickness [8], and turbine position relative to the water-fall [9] on the turbine performance have been explored. The flows through the turbine have also been analyzed [10], [11], [12], [13], [14], [15], [16]. Regarding propeller turbines with simple structures, design methods have been presented [17], [18], [19], [20], [21], turbines successfully mounted in pipe [22], and water supply systems [23] and sewage pipes [24] have been developed. Propeller turbines combined with IoT system have also been presented [25], [26].

Approximately 73% of Japanese islands, which are the main parts of Japan, consist of mountainous terrains. These mountains feature several steep slopes, reaching an altitude of 3000 m in the Chubu region. These islands possess abundant water resources, with an annual precipitation approximately 1.5 times the world average of 1171 mm. Owing to these climatic and geographical characteristics, hydropower generation has been actively conducted in Japan. In a previous report [38], the authors independently pointed out that, among the water resources possessed by the Japanese islands, the regions with abundant technically and economically viable hydro-energy also have significantly higher annual snowfall, reaching approximately 9 m. The authors also identified that small rivers in regions with high snowfall are more likely to have small-scale hydropower plants. Small rivers and irrigation channels in areas with high snowfall frequently carry snow masses during winter months. Microhydraulic turbines installed in these areas suffer from both reduced power generation and operational problems due to snow masses entrained in the rotor, and also damage to the blades. Therefore, developing microhydraulic turbines that can operate at high efficiency while being unaffected by snow masses is crucial for maximizing the year-round application of hydro-energy in regions with heavy snowfall. However, changes in the performance of microhydraulic turbine due to snow masses have never been studied. Therefore, obtaining a design guideline for a microhydraulic turbine that is resistant to snow masses will significantly contribute to the utilization of hydro-energy in snowfall regions worldwide. In a previous study [38], a microhydraulic turbine of an undershot cross-flow type was installed in an irrigation channel in an area with heavy snowfall, and spherical snowballs were released into the water flow toward the turbine to investigate the alterations in the turbine performance. Consequently, the microhydraulic turbine exhibited excellent snowball passability. However, when the snowball diameter exceeded the spacing between the blades, the snowball caught in the rotor decreased the rotor speed or power output. The relationship between the motion of the snowball and the decrease in the rotor performance remains unclear. In addition, when the rotor was stopped by a snowball and then rotated again, the authors observed a temporary increase in the power output compared to clear water (no snowballs); however, the power output after the increase was not measured, and the details remain unknown.

In this study, the same microhydraulic turbine of the undershot cross-flow type as in the previous report [38] was installed in an irrigation channel, and the time variation of the turbine performance was measured when spherical snowballs were released one by one from the upstream. The motion of the snowballs as they passed through the turbine was also observed. Accordingly, the change in the performance could be classified into three modes based on the behavior of the snowballs, which could be organized by the ratio of the snowballs' cross-sectional area to the product of the rotor width and blade interval. Furthermore, the emergence of the power output overshoot phenomenon, in which the power output temporarily increased compared to clear water when the rotor restarts after stopping, was identified, and the relationship between the amount of loss when the rotor stops and the amount of electric energy gained during the overshoot was clarified.

## 2 Irrigation channel and undershot cross-flow hydraulic turbine

### 2.1 Outline of the irrigation channel

The same irrigation channel as in the previous report [38] was utilized for this experiment. Fig. 1 presents the images of the irrigation channel during the non-winter season (May 24, 2018). The irrigation channel is made of U-shaped reinforced concrete and has a width *W* (= 700 mm), a depth *H* (= 700 mm), and a slope of $0.4^{\circ }$. It is located in Shinano-cho, Nagano Prefecture, one of the heaviest snowy regions in Japan. The annual snowfall (1991-2020 average) at the AMeDAS station, located 200 m from the experiment site, is 7.26 m. In this area, snow is observed to accumulate for around 100 days each year. Since December 2016, the authors have independently observed snowfall in this irrigation channel and regularly observed air temperature, water temperature, water level, and flow velocity. The annual mean values of water level and flowrate were 80 mm and 0.06 m^3^/s, respectively.

**Figure 1:** Irrigation channel during no snow season.

Fig. 2 (a) presents the results of snow accretion on the sidewall of the irrigation channel during a snowfall season (January 27, 2018). Some of the snow accretions collapsed toward the irrigation channel after 5 h, as illustrated in Fig. 2 (b).

**Figure 2:** Observation of snow accretion.

Fig. 3 (a) presents the photographs of snow cornices formed on the sidewall of the irrigation channel during snowfall season (February 19, 2018). The snow cornice completely collapsed toward the irrigation channel after 30 min (see Fig. 3 (b)).

**Figure 3:** Observation of cornice.

This type of snow accretion and snow cornice collapse occurs frequently in areas with heavy snowfall depending on weather conditions, such as temperature and wind speed, as well as the amount of snowfall. The action of water currents carries snow masses that drop into irrigation channels down the channels. Therefore, when a microhydraulic turbine is installed in an irrigation channel in a snowy area, snow masses frequently collide with and entangle the turbine blade, thereby deteriorating the power generation owing to low rotor speed and rotor stoppage.

The authors attempt to develop a hydraulic turbine with an output of less than 1 kW. The output is determined from the water depth, water velocity, and channel width. When developing such a hydraulic turbine, it is assumed that the maximum water depth and velocity are approximately 0.3 m and 1 m/s, respectively, and that the channel with is less than 1 m.

### 2.2 Outline of the undershot cross-flow hydraulic turbine

In snowy regions, irrigation channels are relatively narrow, and water flows are often fast even when water levels are low. Consequently, undershot cross-flow-type hydraulic turbines are suitable for generating power from such irrigation channel [13]. In a previous report [38], an undershot cross-flow-type hydraulic turbine was installed in an irrigation channel to investigate changes in power output triggered by snow masses.

In this study, the relationship between the motion of snowballs as they pass through the rotor and the change in the turbine performance is clarified to better understand the performance change owing to snowballs. The same hydraulic turbine as in the previous report [38] was mounted in the irrigation channel described above and utilized in the experiment. An overview is shown in Fig. 4. The rotor diameter *D* and rotor width *B* are 600 mm 300 mm, respectively. A water collector comprising a flat plate is mounted in front of the rotor. It has a length of 380 mm and a straight conduit that is 110 mm long. The width of the inlet of the collector matches the irrigation channel width, and the width of the outlet is 250 mm. The spacing between the rotor tip and irrigation channel bottom is 10 mm. The irrigation channel bottom was slightly modified after the experiment described in the previous paper, and the radius of the inside corner *R* was added at both ends, *R* = 100 mm. Fig. 5 shows an image of the turbine mounted in the irrigation channel, taken from upstream.

**Figure 4:** Geometry and dimensions of the hydraulic turbine of undershot cross-flow type.

**Figure 5:** Image of hydraulic turbine.

Two types of rotors with *n* = 9 and 18 number of blades were tested in the experiment. The objective was to explore the effect of the blade spacing *L* (= πD/n) on the motion of snowballs and the turbine's performance. Fig. 6 shows the geometry and dimensions of the rotor; rotors with *n* = 9 and 18 have L/D values of 0.35 and 0.175, respectively. The inlet angle of blade *β* is 24. In general, there are no recommended values for the rotor diameter *D* and number of blades *n* of an undershot cross-flow-type hydraulic turbine. However, the values of *D* and *n* in this study are approximately equal to those of the rotor presented by Kikuchi et al. [14], which was installed in a 600-mm-wide irrigation channel. The blades have an arc shape, as illustrated in Fig. 7.

**Figure 6:** Rotors used in the experiment.

**Figure 7:** Rotor blade.

## 3 Experimental methods

The permanent-magnet-synchronous-type generator was connected to the rotor-rotating shaft. A load resistor was connected to the generator, and the rotor rotational speed *N* was controlled by varying the resistance $R_{L}$ with $16\;\leq R_{L}\;\leq \;1500\;\Omega$. The output waveform was fed into a PC via an A-D converter, and the value of *N* was calculated by finding the waveform's period of zero crossing. The data sampling frequency was 100 Hz. To express *N* in the nondimensional form, a tip speed ratio of the rotor *λ* is defined as:

(1) $$\lambda =\frac{\pi DN}{60U_{0}}$$

where $U_{0}$ is the flow velocity when the turbine is not installed. The velocity was measured at nine locations in the irrigation channel cross-section $S_{1}$ shown in Fig. 4, by an electromagnetic anemometer, and the mean value was adopted as $U_{0}$.

Effective voltage *V* was calculated using the output waveform of the generator, hence, the power output $P(=3V^{2}/R_{L})$ was obtained. The power output coefficient $C_{p}$, a dimensionless value of *P*, is defined as:

(2) $$C_{p}\;=\frac{P}{0.5\rho_{w}\;H_{0}\;WU_{0}^{3}}$$

where $\rho_{w}$ and $C_{p}$ denote the water density and power generation efficiency, respectively, $H_{0}$ represents the water level at position $S_{1}$ when the turbine is not installed.

To fabricate a spherical snowball, two containers with the shape of a hemispherical shell were filled with snow, and each plane was joined. Fig. 8 shows an image of snowballs with a diameter *d* of 130 mm. From position $S_{2}$, 1000 mm upstream of the water collector, a snowball was released into the water flow, as illustrated in Fig. 4. The snowball was directed downstream toward the turbine. The snowballs were released while the turbine was operating at the rotational speed $N_{0}$, at which the maximum power output $P_{0}$ was obtained in clear water with no snowballs.

**Figure 8:** Snowballs with diameter *d* of 130 mm.

Table 1 summarizes the conditions under which snowballs were released. Experiments were conducted on rotors with *n* = 9 and 18 under six different conditions, from Cases 1 to 6, with the time interval Δ*t* and diameter *d* selected as experimental parameters. In each condition, three snowballs were released, one for each Δ*t*. For Cases 1, 3, and 5, Δ*t* = 5 s, while Δ*t* = 10 s for Cases 2, 4, and 6. In addition, *d* = 130 mm for Cases 1 and 2, *d* = 210 mm for Cases 3 and 4, and *d* = 240 mm for Cases 5 and 6. The average density of the snowballs was 657 kg/m^3^.

**Table 1:** Conditions to release snowball into water flow.

Fig. 9 shows the relative relationship between a 130-mm snowball released into the channel and the turbine rotor. The images were taken using a camera placed 1500 mm upstream from the turbine at 0.5 s (Fig. 9 (a)) and 1 s (Fig. 9 (b)) after the snowball was released. It can be seen that the snowball was near the surface of the water due to buoyancy and was caught in the rotor.

**Figure 9:** Snowball approaching the rotor. Photos taken 0.5 s (a) and 1 s (b) after the release of the snowball.

The water level upstream of the turbine is related to the rotor rotation status, i.e., the power. Therefore, the water level on the channel wall at cross-section $S_{1}$ was read from the video image captured by the camera above, and it determined the time variation of the value $H_{1}$.

In a previous report [38], in addition to the aforementioned camera, a camera located directly above the rotor was utilized to capture images of the upstream and inlet of the rotor to observe the behavior of snowballs. In this study, an endoscope camera (480 × 640 pixels, 25 fps) was installed at the bottom of the channel, 1180 mm upstream from the rotor center axis, to capture an underwater video of the motion of snowballs passing through the turbine and rotor rotation.

## 4 Experimental results and discussion

### 4.1 Turbine performance for clear water

First, the power output characteristics of the turbine were investigated for clear water, i.e., when snowballs were not discharged into the channel. The turbine's power output *P* changes relative to the rotor rotational speed *N*, as shown in Fig. 10. A rotor of *n* = 18 reached a maximum power output of 17.6 *W* at *N* = 36.1 rpm, while a rotor of n = 9 reached a maximum of 15.5 *W* at *N* = 34.1 rpm. At all rotational speeds, the power output of the *n* = 9 case was lower than that of the *n* = 18 case. This is because the rotor with fewer blades received less torque from the water flow. However, at a lower rpm than the maximum efficiency point (*N*≤ 34.1 rpm), the effect of *n* was negligible, and the rotor of *n* = 9 generated the same power as the rotor with *n* = 18. Similar results were obtained in the previous report [38].

**Figure 10:** Relationship between power output *P* and rotor rotational speed *N* for clear water.

The results in Fig. 10 are shown in Fig. 11 for the tip speed ratio *λ* and power coefficient $C_{p}$, with maximum values of 0.164 and 0.186 for *n* = 9 and 18 blades, respectively.

**Figure 11:** Relationship between power coefficient *C*_*p*_ and tip speed ratio *λ* for clear water.

### 4.2 Change in power output owing to a snowball passing through a rotor of *n* = 9

Snowballs were released from upstream toward a rotor of *n* = 9, and the change in the power output *P* was subsequently investigated. The snowballs were released while the turbine was running at $N_{0}$ = 34.1 rpm, the rotational speed at which the maximum power output $P_{0}$ (= 15.5 *W*) was obtained for clear water. Table 2 presents a nondimensional representation of the release conditions summarized in Table 1. The rotor rotational period $T_{0}$ (= 60/$N_{0}$ s) and blade interval *L* for clear water were adopted for the nondimensionalization. The ratio of the snowball mass flowrate $M_{s}$ to the water mass flowrate $M_{w}$ ($M_{s}/M_{w}$) is also included at the bottom of Table 2.

**Table 2:** Nondimensional conditions to release snowball into water flow when *n* = 9.

Fig. 12 shows the time variation of power output with snowball diameter *d* = 130 mm (d/L = 0.62) for Cases 1 (Fig. 12 (A)) and 2 (Fig. 12 (B)), where the snowball release intervals $\Delta t/T_{0}$ were 2.84 and 5.68, respectively. The time of release of the first snowball was set at *t* = 0, and *P* and *t* were expressed in the nondimensional forms by $P_{0}$ and $T_{0}$, respectively. In Case 1, the power output *P* dropped slightly when the second snowball passed through the rotor; however, the difference from the clear water condition was negligible. In Cases 1 and 2, where the diameter of the snowball was smaller than the blade spacing, the snowballs passed smoothly through the rotor without interfering with its rotation. The water level $H_{1}$ upstream of the turbine was not affected by the snowballs (it remained constant).

**Figure 12:** Time variation of power output *P* of rotor of *n* = 9 and *d*/*L* = 0.62 for Case 1 (A) and Case 2 (B).

Fig. 13 shows the change in the power output for d/L = 1, where the diameter of the snowball equals the blade spacing. Case 3 (Fig. 13 (A)) exhibited a temporary drop in the power output at three different times. The time intervals of the power output drops were approximately equal, which is consistent with the snowball release time interval $\Delta t/T_{0}$ = 2.84. The temporary power output drops were triggered by the independent passage of the three snowballs. In Case 4 (Fig. 13 (B)), as in Case 3, a periodic drop in the power output occurred. The power output drops were owing to the passage of the snowballs, and their periods were equal to the release time interval $\Delta t/T_{0}$ = 5.68. The power output minima in Cases 3 and 4 were between 23% and 64% of the power output for clear water. Evidently, when a snowball passed through the rotor, it temporarily interfered with the rotation of the rotor. However, the change in the water level $H_{1}$ upstream of the turbine was minimal.

**Figure 13:** Time variation of power output *P* of rotor of *n* = 9 and *d*/*L* = 1 for Case 3 (A) and Case 4 (B).

The time variation of the power output in Case 5 is presented in Fig. 14 (B) for d/L = 1.15, where the diameter of the snowball was larger than the blade spacing. At $t/T_{0}$ = 2, the power output dropped slightly but recovered in a short time, owing to the first snowball passing through the rotor. The power output then dropped abruptly at $t/T_{0}$ = 4.6 and remained zero for a long time because the rotor stopped rotating because of the entrainment of the second and third snowballs. Then, at $t/T_{0}$ = 25.5, the power output increased rapidly because the rotor resumed rotation, causing all snowballs to flow downstream of the rotor. The power output increased to a maximum of 1.53 times the power output $P_{0}$ for clear water, after which it slowly decreased and approached $P_{0}$. The time variation of the water level $H_{1}$ upstream of the turbine is shown in Fig. 14 (A). The variation of $H_{1}/H_{10}$ is made dimensionless by the water level $H_{10}$ at clear water. $H_{1}$ began to increase at $t/T_{0}$ = 4.6. This is because the stopped rotor by the snowballs interfered with the water flow in the channel. Finally, it reached a maximum value of 1.22 $H_{10}$ at $t/T_{0}$ = 20.5. The water level increased, and immediately after the rotor re-rotated, the flowrate of water into the rotor temporarily increased compared to clear water, thereby resulting in a higher power output than that of clear water, as described above. Thereafter, as $H_{1}$ approached the clear water value $H_{10}$, the power output gradually decreased to the clear water value. A previous report [38] also observed *P* exceeding $P_{0}$. However, in the previous report, the measurement was terminated immediately after *P* exceeded *P*; therefore, the comprehensive details of the *P* overshoot phenomenon were revealed for the first time in this study. In Case 6, which corresponds to a time variation twice as long as that in Case 5, the same power output variation as in Case 5 was observed, as shown in Fig. 14 (C). The power output decreased, recovered for a short time, and then stopped at $t/T_{0}$ = 12.7. Then, it recovered slightly, stopped again, and then increased sharply at $t/T_{0}$ = 17.3. Thereafter, an overshoot phenomenon appeared owing to the rising water level upstream of the turbine.

**Figure 14:** Time variations of the water level *H*_1_ upstream of the turbine for Case 5 (A) and power output *P* of rotor of *n* = 9 and *d*/*L* = 1.15 for Case 5 (B) and Case 6 (C).

### 4.3 Change in power output owing to snowball passing through a rotor of n = 18

The change in power output *P* owing to snowballs were investigated for the rotor of *n* = 18 blades. Snowballs were released at the rotational speed $N_{0}$ = 36.1 rpm, at which the maximum power output $P_{0}$ = 17.6 *W* was generated for clear water. Table 3 presents the experimental conditions expressed in the dimensionless form.

**Table 3:** Nondimensional conditions to release snowball into water flow when *n* = 18.

Fig. 15 shows the results for d/L = 1.24, where the diameter of the snowball was slightly larger than the blade spacing. The power output and time were nondimensionalized, as in the case *n* = 9. In Case 1 (Fig. 15 (A)), where the snowball release time interval $\Delta t/T_{0}$ = 3.01, the power output decreased periodically. The nondimensional period coincided with $\Delta t/T_{0}$. The periodic decrease was owing to the three snowballs passing through the rotor independently. In Case 2 (Fig. 15 (B)), with $\Delta t/T_{0}$ = 6.02, the power output decreased periodically, as in Case 1. Its nondimensional period was equal to $\Delta t/T_{0}$. The periodic variation was similar to the results of Cases 3 and 4 for rotors with *n* = 9, as shown in Fig. 13. The change in the water level $H_{1}$ upstream of the turbine was similarly small.

**Figure 15:** Time variation of power output *P* of rotor of *n* = 18 and *d*/*L* = 1.24 for Case 1 (A) and Case 2 (B).

The time variation of power output *P* for d/L = 2 with increasing snowball diameter is shown in Fig. 16. In Case 3 (Fig. 16 (A)) with $\Delta t/T_{0}$ = 3.01, *P* dropped abruptly at $t/T_{0}$ = 2.8 and remained at P=0 until $t/T_{0}$ = 19.3. Three snowballs stopped the rotor rotation. Then, at $t/T_{0}$ = 19.3, the power output increased rapidly, reaching 1.55 times the value of $P_{0}$ for clear water, owing to the three snowballs flowing downstream of the rotor. After reaching its maximum value, the power output gradually decreased over time, approaching $P_{0}$. This overshooting of *P* is due to the rising water level, as shown in Fig. 14. Case 4 (Fig. 16 (B)), with $\Delta t/T_{0}$ = 6.02, produced time variations similar to those in Case 3.

**Figure 16:** Time variation of power output *P* of rotor of *n* = 18 and *d*/*L* = 2 for Case 3 (A) and Case 4 (B).

Fig. 17 shows the time variation of *P* for a further increase in the snowball diameter, d/L = 2.3, and for Cases 5 (Fig. 17 (A)) and 6 (Fig. 17 (B)), $\Delta t/T_{0}$ = 3.01 and 6.02, respectively. The time variations were similar to those shown in Fig. for Cases 3 and 4. The maximum values of *P* in Cases 5 and 6 during overshoot are 1.65 and 1.82, respectively, which are slightly higher than the maximum values shown in Fig. 16 for Cases 3 and 4. This is because the snowball diameter was larger than the blade spacing; hence, the snowball caught in the rotor cannot flow out smoothly, thereby resulting in a longer rotor stoppage time.

**Figure 17:** Time variation of power output *P* of rotor of *n* = 18 and *d*/*L* = 2.3 for Case 5 (A) and Case 6 (B).

### 4.4 Relationship between time variation in power output and snowball behavior

The time variation modes of power output described above are classified into three types. First, Variation A is the variation of Cases 1 and 2 for *n* = 9, shown in Fig. 12, where the effect of snowballs hardly appears. Variation A also includes the variation of Cases 3 and 4 for *n* = 9, shown in Fig. 13, and that of Cases 1 and 2 for *n* = 18, shown in Fig. 15, where the power output is periodically affected by snowballs. Second, Variation B is the variation of Cases 5 and 6 for *n* = 9, shown in Fig. 14, where some snowballs stop their power output for a certain time. Third, Variation C is the variation of Cases 3 and 4 for *n* = 18, shown in Fig. 16, and that of Cases 5 and 6 for *n* = 18, shown in Fig. 17, where all snowballs stop the power output for a certain time.

An endoscope camera fixed to the bottom of the channel upstream of the rotor was utilized to record the video of the snowball and rotor. The time when the power output exhibited a characteristic change was selected, and still images were extracted. As Variation A, considering Case 1 as an example with *n* = 18 and d/L = 1.24 in Fig. 15, three images at three different times were selected, as illustrated in Fig. 18. Fig. 18 also includes an illustration of a rotor and snowball extracted from the image. The red lines in the image indicate the blade leading and trailing edges, which are connected by lines to the blades in the illustration. Fig. 15 also clearly presents the time of the image. In Variation A, three snowballs emitted in succession pass through the rotor independently and exhibit a periodic drop in the power output of the same magnitude. Therefore, the authors focused on the motion of the third snowball. Fig. 18 (a) shows the nondimensional time $t/T_{0}$ = 7.74, when the snowball reached the inlet of the rotor. Immediately after this, at $t/T_{0}$ = 7.77, the snowball flowed downstream until just before it was engulfed by the rotor, as shown in Fig. 18 (b). Fig. 18 (c) shows the time when the snowball was entrained between the blades ($t/T_{0}$ = 7.79). These three times correspond to just before the turbine's power output temporarily drops abruptly, as shown in Fig. 15. Therefore, the snowballs between the blades shown in Fig. 18 (c) came into contact with the bottom of the channel as the rotor rotates, and the negative torque (torque preventing the rotor from rotating forward) caused by the frictional force acts on the rotor, temporarily decreasing the rotor rotational speed or power output.

**Figure 18:** Relative positional relation between snowballs and rotor for Variation A (Case 1 of *n* = 18) at *t*/*T*_0_ = 7.74 (a), *t*/*T*_0_ = 7.77 (b), and *t*/*T*_0_ = 7.79 (c).

Fig. 19 shows the snowball and rotor for Case 5 with *n* = 9 and d/L = 1.15, classified as Variation B. The change in the power output is similar to that shown in Fig. 14. Fig. 19 (a) shows the image at $t/T_{0}$ = 1.1, just before the first snowball flowed into the rotor. This snowball was immediately entrained between the blades at $t/T_{0}$ = 1.14, as shown in Fig. 19 (b), and then flowed downstream of the rotor. The entrainment and outflow of the first snowball induced a temporary drop in the power output at $t/T_{0}$ = 2, as shown in Fig. 14. At $t/T_{0}$ = 3.94, a second snowball was just before the rotor (Fig. 19 (c)). At $t/T_{0}$ = 6.81, the snowball began to roll into the rotor (Fig. 19 (d)). Simultaneously, the third snowball reached just before the rotor and made contact with the second snowball that precedes it. At this time, the power output was zero, as shown in Fig. 14. It can be seen that the second snowball, caught between the blades and channel bottom, stopped the rotor rotation. As time passed, the second snowball was crushed by the shearing action of the blades, the rotor rotated at a very low speed to discharge the crushed snowball downstream, and at $t/T_{0}$ = 22.7, the third snowball was entrained into the rotor (Fig. 19 (e)). After the third snowball was discharged downstream of the rotor, the power output increased rapidly at $t/T_{0}$ = 25.9.

**Figure 19:** Relative positional relation between snowballs and rotor for Variation B (Case 5 of *n* = 9) at *t*/*T*_0_ = 1.1 (a), *t*/*T*_0_ = 1.14 (b), *t*/*T*_0_ = 3.94 (c), *t*/*T*_0_ = 6.81 (d), and *t*/*T*_0_ = 22.7 (e).

Fig. 20 shows the snowballs and rotor in Case 5 with *n* = 18 and d/L = 2.3, classified as Variation C. The time variation of the power output is shown in Fig. 17. The first snowball was just before the rotor at $t/T_{0}$ = 1.78, as shown in Fig. 20 (a). This snowball was entrained into the rotor at $t/T_{0}$ = 5.43 (Fig. 20 (b)). This entrainment caused the power output to stop, as shown in Fig. 17. Simultaneously, the second snowball approached the rotor entrance and was in series with the first snowball; at $t/T_{0}$ = 10.3, the first and second snowballs were entrained in the rotor, and the third snowball was just before the rotor, as shown in Fig. 20 (c). Later, at $t/T_{0}$ = 13.3 and 16.9, the first snowball flowed downstream of the rotor; however, the second snowball remained entrained, and the third snowball was stationary just before the rotor, as shown in Figs. 20 (d) and (e), respectively. At $t/T_{0}$ = 27.8, the second snowball also flowed downstream of the rotor; however, the third snowball became entrained, as shown in Fig. 20 (f). Variation C caused the rotor to stop rotating for a certain period of time; hence, the power output stopped for a long time.

**Figure 20:** Relative positional relation between snowballs and rotor for Variation C (Case 5 of *n* = 18) at *t*/*T*_0_ = 1.78 (a), *t*/*T*_0_ = 5.43 (b), *t*/*T*_0_ = 10.3 (c), *t*/*T*_0_ = 13.3 (d), *t*/*T*_0_ = 16.9 (e), and *t*/*T*_0_ = 27.8 (f).

The conditions for the appearance of Variations A, B, and C were investigated. As described above, snowballs were entrained between the blades and channel bottom, causing a change in the power output. The dependence of this entrainment on the blade interval *L* was reported in the previous paper [38]. In Variations B and C, the snowballs lodged at the rotor inlet reduced the effective area of the inlet. The ratio of the cross-sectional area $\pi {\left(d/2\right)}^{2}$ of one snowball to the product *BL* of the rotor width *B* (=300 mm) and *L*, $\pi {\left(d/2\right)}^{2}/BL$, on the horizontal axis, and the release time interval $\Delta t/T_{0}$ on the vertical axis, the release conditions for *n* = 9 and 18, are shown in Fig. 21. Variation A appears for $\pi {\left(d/2\right)}^{2}/BL\leq 0.551$, thus indicating that the horizontal axis adequately expresses the effect of *n* on the appearance of Variation A, while the conditions for *n* = 9 and 18 are mixed. However, it does not depend on the value of $\Delta t/T_{0}$ on the vertical axis. Variation C appears for $\pi {\left(d/2\right)}^{2}/BL\geq 1.1$. This is owing to the large snowball diameter. Variation B exists between Variations A and C. The horizontal axis appropriately classifies Variation B, where the characteristics of Variations A and C coexist. Hence, the three characteristic time variations of the power output can be organized by the ratio of the cross-sectional area of the snowball to the area between the blades.

**Figure 21:** Map of changes in power output for Variation A, Variation B, and Variation C.

### 4.5 Decrease and increase in electric power generation due to snowballs

As shown in Figure 14, Figure 16, Figure 17, the power output *P* of Variations B and C remained at zero, then rapidly increasing until it reached a maximum value exceeding $P_{0}$ for clear water, and then gradually decreased toward $P_{0}$. To examine the electric energy produced by this overshooting phenomenon, the electric energy was calculated based on the time variation of *P* for Variations B and C. The ratio of the electric energy that increases due to the overshoot phenomenon, $E_{+}$, to the electric energy lost due to the snowball, $E_{-}$, is defined as the electric energy recovery rate $\overset{ˆ}{E}$ as expressed in Eq. (3) (the details of $E_{-}$ and $E_{+}$ are expressed in Eq. (4)).

(3) $$\overset{ˆ}{E}=E_{+}/E_{-}$$

(4) $$E_{-}\;=\int_{t1}^{t2}(P-P_{0})\;dt,E_{+}\;=\int_{t3}^{t4}(P-P_{0})\;dt$$

where $t_{1}$ and $t_{2}$ represent the start and end times of P=0, respectively; t3 and t4 denote the times when *P* overshoots and exceeds the power output $P_{0}$ at clear flow and returns to $P_{0}$, respectively.

Table 4 shows the $\overset{ˆ}{E}$ values for Variations B and C. Note that Variation B is the result of Cases 5 and 6 for *n* = 9, and Variation C is the result of Cases 3-6 for *n* = 18. For Variation C, 53%-65% of the electric energy lost during rotor stoppage is recovered during overshoot. This is because the long rotor stoppage time and large number of blades caused the high damming effect to persist for a long time, thereby leading to a increase in the water level and a large overshoot. The difference in $\overset{ˆ}{E}$ values between Cases 3 and 6 is negligible, and the effect of the snowball diameter and release time interval, i.e., the mass flowrate of snowballs, is negligible. The absolute value of $\overset{ˆ}{E}$ for Variation B is smaller than that for Variation C. This is especially true for Case 6, where the rotor stop time is short but does not result in a large overshoot.

**Table 4:** Recovery rate of electric energy $\overset{ˆ}{E}$.

## 5 Conclusion

To maximize the year-round utilization of hydro-energy in the channels of regions with heavy snowfall, it is crucial to develop a microhydraulic turbine that can generate electricity even in channels where snow masses are flowing downstream. In a previous paper, an undershot cross-flow-type hydraulic turbine was installed in an irrigation channel in such a region to examine the changes in the performance due to spherical snowballs flowing from upstream. In this study, a hydraulic turbine of an undershot cross-flow type was mounted in an irrigation channel, and spherical snowballs were released successively at regular time intervals from upstream. The turbine's power output was measured, and the behavior of the snowballs was captured on video using multiple cameras. Accordingly, the following conclusions were obtained:

(1) The change in turbine performance owing to snowballs can be classified into Variations A, B, and C. In Variation A, the turbine power output remained unchanged or decreased periodically from the maximum power output for clear water. In Variation B, some snowballs caused the turbine power output to drop to zero for a certain period. Finally, in Variation C, the turbine power output decreased to zero for a certain period for all snowballs.
(2) Variations A, B, and C appear according to the ratio to the product of the rotor width and blade interval. The variations do not depend on the release time interval of the snowballs.
(3) The turbine power output in Variations B and C continued to be zero, then rapidly increased, thereby reaching a maximum value above the maximum power output, and gradually decreased toward the maximum power output. In other words, an overshoot phenomenon in the power output appears immediately after the rotor is stopped by a snowball and then rotates again. The overshoot phenomenon is triggered by the rising water level upstream of the turbine that occurs when the rotor stops.
(4) The ratio of the excess electric energy gained during overshoot to the electric energy lost during the rotor stoppage, or the electric energy recovery rate $\overset{ˆ}{E}$, is 0.53 $\leq \overset{ˆ}{E}\leq$ 0.65 for Variation C. However, the effect of the diameter of the snowball and release time interval of the snowball, i.e., the mass flowrate of the snowball, on $\overset{ˆ}{E}$ is negligible.

## CRediT authorship contribution statement

**Eiichi Satou:** Conceptualization, Data curation, Formal analysis, Supervision, Validation, Visualization, Writing – original draft, Writing – review & editing. **Tomomi Uchiyama:** Conceptualization, Data curation, Formal analysis, Validation, Visualization, Writing – original draft, Writing – review & editing. **Kotaro Takamure:** Conceptualization, Data curation, Formal analysis, Validation, Visualization, Writing – original draft, Writing – review & editing. **Toshihiko Ikeda:** Conceptualization, Data curation, Formal analysis, Validation, Visualization, Writing – original draft, Writing – review & editing. **Tomoko Okayama:** Conceptualization, Data curation, Formal analysis, Validation, Visualization, Writing – original draft, Writing – review & editing. **Tomoaki Miyazawa:** Conceptualization, Data curation, Formal analysis, Validation, Visualization, Writing – original draft, Writing – review & editing. **Daisuke Tsunashima:** Conceptualization, Data curation, Formal analysis, Validation, Visualization, Writing – original draft, Writing – review & editing.

## Declaration of Competing Interest

The authors declare that they have no known competing financial interests or personal relationships that could have appeared to influence the work reported in this paper.

## Data Availability

Data will be made available on request.

## References

[1] Vagnonia E., Andolfatto L., Richard S., Munch-Alligne C., Avellana F. (2018). Hydraulic performance evaluation of a micro-turbine with counter rotating runners by experimental investigation and numerical simulation. Renew. Energy.

[2] Williamson S.J., Stark B.H., Booker J.D. (2014). Low head pico hydro turbine selection using a multi-criteria analysis. Renew. Energy.

[3] Loots I., Dijk M., van Barta B., Vuuren S.J., van Bhagwan J.N. (2015). A review of low head hydropower technologies and applications in a South African context. Renew. Sustain. Energy Rev..

[4] McNabola A., Coughlan P., Corcoran L., Power C., Williams A.P., Harris I., Gallagher J., Styles D. (2014). Energy recovery in the water industry using micro-hydropower: an opportunity to improve sustainability. Water Policy.

[5] Al-Shetwi A.Q. (2022). Sustainable development of renewable energy integrated power sector: trends, environmental impacts, and recent challenges. Sci. Total Environ..

[6] Du J., Ge Z., Hao W., Shi X., Yuan F., Yu W., Wang D., Yang X. (2022). Study on the effects of runner geometric parameters on the performance of micro Francis turbines used in water supply system of high-rise buildings. Energy.

[7] Choi Y.-D., Lim J.I., Kim Y.-T., Lee Y.H. (2008). Performance and internal flow characteristics of a cross-flow hydro turbine by the shapes of nozzle and runner blade. J. Fluid Sci. Technol..

[8] Yamazaki M., Oike S., Iio S., Ikeda T. (2011). Proc. 11th Int. Sympo. Fluid Power.

[9] Katayama Y., Iio S., Veerapun S. (2014). Effect of runner position on performance for open type cross-flow turbine utilizing waterfalls. Int. Rev. Mech. Eng. J..

[10] Nishi Y., Inagaki T., Li Y., Omiya R., Hatano K. (2014). The flow field of undershot cross-flow water turbines based on PIV measurements and numerical analysis. Int. J. Fluid Mach. Syst..

[11] Nishi Y., Inagaki T., Li Y., Omiya R., Fukutomi J. (2014). Study on an undershot cross-flow water turbine. J. Therm. Sci..

[12] Uchiyama T., Uehara S., Fukuhara H., Iio S., Ikeda T. (2015). Numerical study on the flow and performance of an open cross-flow mini-hydraulic turbine. Proc. Inst. Mech. Eng. A, J. Power Energy.

[13] Uchiyama T., Mizoguchi S., Iio S., Katayama Y., Ikeda T. (2016). Effects of clearance between rotor and ground on the performance of an open cross-flow-type nano-hydraulic turbine. J. Energy Power Eng..

[14] Kikuchi Y., Kiwata T., Watada S., Kono T. (2018). Experimental study on performance of undershot water wheel in snow drainageway at Shiramine district by field test. Adv. Exp. Mech..

[15] Shikama H., Wang T., Yamagata T., Fujisawa N. (2021). Experimental and numerical studies on the performance of a waterfall-type cross-flow hydraulic turbine. Energy Sustain. Dev..

[16] Mehr G., Durali M., Khakrand M.H., Hoghooghi H. (2021). A novel design and performance optimization methodology for hydraulic Cross-Flow turbines using successive numerical simulations. Renew. Energy.

[17] Alexandera K.V., Giddensb E.P., Fullera A.M. (2009). Axial-flow turbines for low head microhydro systems. Renew. Energy.

[18] Singh P., Nestmann F. (2011). Experimental investigation of the influence of blade height and blade number on the performance of low head axial flow turbines. Renew. Energy.

[19] Ferro L.M.C., Gato L.M.C., Falcao A.F.O. (2011). Design of the rotor blades of a mini hydraulic bulb-turbine. Renew. Energy.

[20] Sotoude M.H., Mirghavami S.M., Chini S.F., Riasi A. (2019). Developing a method to design and simulation of a very low head axial turbine with adjustable rotor blades. Renew. Energy.

[21] Tran B.N., Jeong H., Kim J.-H., Park J.-S., Yang C. (2020). Effects of tip clearance size on energy performance and pressure fluctuation of a tidal propeller turbine. Energies.

[22] Samora I., Hasmatuchi V., Munch-Alligne C., Franca M.J., Schleiss A.J., Ramosa H.M. (2016). Experimental characterization of a five blade tubular propeller turbine for pipe inline installation. Renew. Energy.

[23] Du J., Yang H., Shen Z., Chen J. (2017). Micro hydro power generation from water supply system in high rise buildings using pump as turbines. Energy.

[24] Uchiyama T., Honda S., Degawa T. (2018). Development of a propeller-type hollow micro hydraulic turbine with excellent performance in passing foreign matter. Renew. Energy.

[25] Uchiyama T., Takamure Y., Okuno K., Sato E. (2021). Development of a self-powered wireless sensor node to measure the water flowrate by using a turbine flowmeter. Int. Things.

[26] Takamure K., Uchiyama T., Horie K., Nakayama H. (2022). Enhancing effect of cone on efficiency of a self-powered IoT-based hydro turbine. Adv. Mech. Eng..

[27] Nakajima M., Iio S., Ikeda T. (2008). Performance of Savonius rotor for environmentally friendly hydraulic turbine. J. Fluid Sci. Technol..

[28] Golecha K., Eldho T.I., Prabhu S.V. (2011). Influence of the deflector plate on the performance of modified Savonius water turbine. Appl. Energy.

[29] Iio S., Katayama Y., Uchiyama F., Sato E., Ikeda T. (2011). Influence of setting condition on characteristics of Savonius hydraulic turbine with a shield plate. J. Therm. Sci..

[30] Uchiyama T., Gu Q., Degawa T., Iio S., Ikeda T., Takamure K. (2020). Numerical simulations of the flow and performance of a hydraulic Savonius turbine by the vortex in cell method with volume penalization. Renew. Energy.

[31] Takamure K., Wang H., Uchiyama T., Iio S., Ikeda T. (2021). Vortex-in-cell simulation of the flow and performance of a Savonius hydraulic turbine with S-shaped blades. J. Renew. Sustain. Energy.

[32] Antheaume S., Maitre T., Achard J.-L. (2008). Hydraulic Darrieus turbines efficiency for free fluid flow conditions versus power farms conditions. Renew. Energy.

[33] Talukdar P.K., Kulkarni V., Saha U.K. (2018). Field-testing of model helical-bladed hydrokinetic turbines for small-scale power generation. Renew. Energy.

[34] Yosry A.G., Fernandez-Jimenez A., Alvarez-Alvarez E., Marigorta E.B. (2021). Design and characterization of a vertical-axis micro tidal turbine for low velocity scenarios. Energy Convers. Manag..

[35] Ikeda T., Iio S., Tatsuno K. (2010). Performance of nano-hydraulic turbine utilizing waterfalls. Renew. Energy.

[36] Uchiyama T., Fukuhara H., Iio S., Ikeda T. (2013). Numerical simulation of water flow through a nano-hydraulic turbine of waterfall-type by particle method. Int. J. Rotating Mach..

[37] Elgammi M., Hamad A.A. (2022). A feasibility study of operating a low static pressure head micro pelton turbine based on water hammer phenomenon. Renew. Energy.

[38] Satou E., Ikeda T., Uchiyama T., Okayama T., Miyazawa T., Takamure K., Tsunashima D. (2022). Development of an undershot cross-flow hydraulic turbine resistant to snow and ice masses flowing in an installation channel. Renew. Energy.

